# Improvement of self‐administration experience with a new injection device: Real‐life experience with risankizumab in patients with psoriasis

**DOI:** 10.1111/srt.13902

**Published:** 2024-08-20

**Authors:** Alexandra Maria Giovanna Brunasso, Ilaria Salvi, Stefania Sorbara, Andrea Muracchioli, Elena De Col, Manuela Baldari, Aurora Parodi, Emanuele Cozzani, Martina Burlando

**Affiliations:** ^1^ Unit of Dermatology Villa Scassi Hospital ASL3 Genoa Italy; ^2^ Section of Dermatology Department of Health Sciences (DiSSal) University of Genoa Genoa Italy; ^3^ IRCCS San Martino University Hospital Genoa Italy; ^4^ Division of Dermatology EO Galliera Genoa Italy; ^5^ Unit of Dermatology San Bartolomeo Hospital La Spezia Italy; ^6^ Unit of Dermatology Civil Hospital of Imperia Imperia Italy; ^7^ Unit of Dermatology Civil Hospital of Sestri Levante Sestri Levante Genoa Italy

**Keywords:** biologic treatment, dermatology, needle phobia, psoriasis, risankizumab, trypanophobia

## Abstract

**Background:**

Trypanophobia or “needle phobia” represents a potential hindrance to the effective management of chronic diseases whenever an injectable therapy might be required, especially in case of frequent administrations. Psoriasis, a chronic dermatologic disease, can be effectively treated with biologic drugs administered subcutaneously. Thankfully, anti‐IL‐23 drugs require few administrations per year and are available in prefilled pens that hide the needle, thus representing a convenient option in patients with trypanophobia.

**Methods:**

An observational multicentric study was conducted on patients with moderate‐to‐severe psoriasis who were treated with 75 mg × 2 risankizumab prefilled syringe therapy for more than 6 months and reported a loss of efficacy measured by the Psoriasis Area and Severity Index (PASI) from PASI 90 to PASI 75 attributed to a reduction of adherence due to trypanophobia. The patients were switched to 1 prefilled pen of risankizumab 150 mg and asked to fill out the Self‐Injection Assessment Questionnaire (SIAQ) before and after the injection at week 0 and at the following administration after 12 weeks. Subjects scored each item of the SIAQ on a 5‐point scale, scores were later transformed from 0 (worst experience) to 10 (best experience).

**Results:**

Twenty‐two patients were enrolled. The mean SIAQ predose domain scores were 5.5 for feelings about injection, 6.2 for self‐confidence, and 6.4 for satisfaction with self‐injection. After dose scores were higher (> 8.5) for each of the six domains at Week 0 and even higher after 12 weeks (> 9.0).

**Conclusions:**

User‐friendly devices, such as prefilled pens, and a lower number of injections improved patient satisfaction in a group of patients with psoriasis on treatment with biologic drugs. We believe that treatment adherence could be positively influenced by such changes in the way of administration of a biologic treatment.

## 1 INTRODUCTION

Trypanophobia or “needle phobia” is a common problem that affects many people, with an estimated prevalence of 20%–50% in adolescents and 20%–30% in adults. Although its prevalence tends to decrease with age, it remains an important issue to address in clinical practice.^1^ Patients suffering from chronic diseases may require injectable therapy. However, the fear of needles might impede proper treatment, leading to serious health consequences due to noncompliance with medical care.^1^, ^2^

Psoriasis is a chronic illness affecting millions worldwide.^3^ Fortunately, biologic drugs can effectively manage the symptoms of this disease. However, some patients fear an injection‐based treatment, especially when it requires frequent administrations. Moreover, patients who achieve clinical remission are less motivated to adhere to their treatment plan. Skipping or delaying the injections due to trypanophobia can negatively impact drug survival rates.^3^

It is noteworthy that anti‐tumor necrosis factor (TNF) therapies require frequent administration (bi‐weekly, weekly, or every other week), whereas anti‐interleukin 17 (IL‐17) treatments are typically administered every 4 weeks. Anti‐IL‐23 drugs have a reduced schedule (every 8 to 12 weeks) of administration. The advantage of biologicals consists of prefilled syringes or pens hiding the needle. Such devices represent a good option for patients who are afraid of needles.^4^

The aim of our study is to evaluate, using the Self Injection Assessment Questionnaire (SIAQ) the benefits of Risankizumab prefilled 150‐mg pen, identifying any psychological or social barriers that may prevent patients from following their injection schedule.^5^

## 2 METHODS AND MATERIALS

Between July 2023 and September 2023, a study was conducted on patients diagnosed with moderate‐to‐severe psoriasis who were treated with risankizumab prefilled syringe therapy for more than 6 months and reported a loss of efficacy measured by the Psoriasis Area and Severity Index (PASI) from PASI 90 to PASI 75 for a reduction of adherence due to fear of injections. The study included patients who were at least 18 years old, able to understand informed consent, and eligible for systemic biologic therapy.

During the study, patients stopped self‐administering the 75 mg × 2 prefilled injections and were switched to 1 prefilled pen of risankizumab 150 mg. They were asked to fill out the Self‐Injection Assessment Questionnaire (SIAQ) before and after the procedure, as well as after 12 weeks. Demographic characteristics such as age, sex, duration of psoriasis, and history of systemic therapies were recorded. Additionally, the presence of depression, whether the patient was a naive patient or had undergone previous biologic therapy, was also noted.

The SIAQ is divided into a premodule and a postmodule.^6^ The premodule is given to the patient immediately before the injection at Week 0 and includes three domains: “feelings about injections,” “self‐confidence,” and “satisfaction with self‐injection.” The postmodule is completed by the patient 20–40 min after each injection at Weeks 0 and 12. The postmodule comprises six domains: “feelings about injections,” “self‐image,” “self‐confidence,” “pain and skin reactions during or after the injection,” “ease of use of the self‐injection device,” and “satisfaction with self‐injection.” Each domain consists of several individual questions with scores ranging from 1 to 5, which are later transformed into scores ranging from 0 (worst experience) to 10 (best experience). Higher domain scores indicate higher acceptability by patients to use the prefilled injection.^6^ Four Ligurian dermatology outpatient psoriasis clinics conducted the study.

The descriptive statistics used in the data analysis included the frequencies and proportions for the categorical variables. This helped identify the number of observations that fell into each category and the proportion of the total observations each category represented. The mean and standard deviation were reported for continuous, nonnormally distributed variables. The mean value was used to determine the central tendency of the data, while the standard deviation indicated the degree of variability of the data around the mean. This detailed statistical analysis helped to provide a comprehensive understanding of the data and its characteristics.

## 3 RESULTS

Twenty‐two psoriatic patients, 12 males and 10 females, were enrolled. The average age of patients was 63 years, and the average disease duration was 19.7 years, with a mean duration of systemic therapy of 7.4 years. Ten patients had previous experience with biologics other than risankizumab. Six out of 22 (27.3%) of the patients had a history of depression.

The study evaluated the patients' experience with self‐injection using a prefilled pen. The mean SIAQ predose (3 modules) domain scores were 5.5 for feelings about injection, 6.2 for self‐confidence, and 6.4 for satisfaction with self‐injection. Postdose (6 modules) domain scores were higher (> 8.5) for each domain at Week 0 and even higher after 12 weeks (> 9.0) (Figure 1).

**FIGURE 1:** Results for the three domains “feelings about injections,” “self‐confidence,” and “satisfaction with self‐injection” at different time points.

The SIAQ included several questions to evaluate specific aspects of the self‐injection process. When asked about the self‐injection device's difficulty, 20/22 (90.9%) of patients found it “easy” or “very easy” at Week 0, followed by 21/22 (95.5%) at Week 12. Similarly, 90.9% of patients found it “easy” or “very easy” to self‐administer the injection without any help at Week 0, followed by 95.5% at Week 12. Additionally, 95.5% of patients found it “very easy” or “extremely easy” to give themselves an injection at Week 0, followed by 19/22 (86,4%) at Week 12. Furthermore, 90.9% of the patients were “satisfied” or “very satisfied” with their current method of taking medication (self‐injection).

The study also analyzed the relationship between the patient's duration of systemic therapy and disease duration with their SIAQ scores. The results showed that patients who had been on systemic therapy for more than 7 years had lower SIAQ predose domain scores, while patients with disease duration of more than 19 years had higher predose domain scores, both in line with the mean score. However, these differences were not statistically significant (*p* > 0.05). Patients with depressive symptoms had lower SIAQ predose domain scores than the mean values, but the difference was not significant in the post‐SIAQ scores after 0 and 12 weeks (*p* > 0.05).

## 4 DISCUSSION

Needle phobia is a medical condition that affects at least 20% of the population.^1^ People with needle phobia tend to avoid medical care, which hinders the quality and timeliness of the health care they receive. Nowadays, the most effective treatments for psoriasis are administered as subcutaneous injections, which might discourage patients suffering from psoriasis and needle phobia from administrating therapy, leading to severe consequences for their health.^2^

Less‐frequent treatment regimens (as with IL‐23 blockers) and the introduction of prefilled pens that hide the needle could make self‐administration less intimidating. In Italy, for instance, the risankizumab 150 mg prefilled pen has been available for about a year, replacing the two prefilled 75 mg syringes previously available. The new device has been positively received by patients who were already receiving the anti‐IL‐23 therapy due to the reduction of injections, preventing loss of adherence due to needle phobia, which resulted in a loss of treatment effectiveness.

This study indicates how even patients with severe needle phobia, who were previously more likely to face a loss of drug efficacy due to reduced adherence, can benefit from a pen device. SIAQ scores before the first injection were on average lower than the following ones: this reflects the patients’ fear deriving from previous treatments. After injection, the SIAQ score increased for every patient, indicating that the new device inspired confidence, particularly after 12 weeks. Patients with a long history of systemic therapy had lower than average initial SIAQ values because they had been injecting for years, resulting in a greater fear of needles or impatience with needles that seems to diminish when switching to the self‐injector.

In patients with a long duration of the disease, the SIAQ value was higher than average, indicating that even needle‐phobic patients can be willing to perform injections in order to receive systemic therapy when they perceive they need it. However, the problem arises when needle‐phobic patients autonomously avoid the injections after achieving clinical remission, leading to a potential loss of treatment effectiveness.

Although these data were not statistically significant, patients with self‐reported depressive syndrome had lower SIAQ scores at baseline, but their scores increased in the following appointments. This finding confirms that the fear of needles is a significant issue in patients who have already undergone systemic injection therapies. The marketing of automatic devices capable of hiding the needle, which is less painful, makes a significant contribution in terms of therapeutic adherence.

The study has some limitations, including the small number of patients selected and the absence of a control group. However, it highlights the importance of recognizing needle phobia, which is often overlooked by doctors. If not managed, needle phobia can lead to poor therapeutic adherence and a possible recurrence of the disease.^7^

## 5 CONCLUSION

This study provides fascinating insights. It reveals that the loss of effectiveness of a therapy may not be caused by the drug itself, but rather by patients' fear of needles, which leads to the avoidance of administration. Understanding this could enable us to make some changes to our strategies to improve adherence.

## CONFLICT OF INTEREST STATEMENT

The authors declare no conflicts of interest.

## CONSENT STATEMENT

Informed consent was obtained from all subjects involved in the study.

## Data Availability

The data that support the findings of this study are available on request from the corresponding author. The data are not publicly available due to privacy or ethical restrictions.
